The article "Silencing of APE1 Enhances Sensitivity of Human Hepatocellular Carcinoma Cells to Radiotherapy In Vitro and in a Xenograft Model" was retracted in 2023. Reasons: errors in the images; duplicated images; overlap with earlier publications; original data or images not available.

# Silencing of APE1 Enhances Sensitivity of Human Hepatocellular Carcinoma Cells to Radiotherapy *In Vitro* and in a Xenograft Model

**DOI:** 10.1371/journal.pone.0055313

**Published:** 2013-02-13

**Authors:** Yanping Cun, Nan Dai, Chengjie Xiong, Mengxia Li, Jiangdong Sui, Chengyuan Qian, Zheng Li, Dong Wang

**Affiliations:** 1 Cancer Center, Daping Hospital and Research Institute of Surgery, Third Military Medical University, Chongqing, People’s Republic of China; 2 Department of Orthopedics, Xinqiao Hospital, Third Military Medical University, Chongqing, People’s Republic of China; University of Maastricht (UM), The Netherlands

## Abstract

Resistance to radiotherapy is a key limitation for the treatment of human hepatocellular carcinoma (HCC). To overcome this problem, we investigated the correlation between radioresistance and the human apurinic/apyrimidinic endonuclease (APE1), a bifunctional protein, which plays an important role in DNA repair and redox regulation activity of transcription factors. In the present study, we examined the radiosensitivity profiles of three human HCC cell lines, HepG2, Hep3B, and MHCC97L, using the adenoviral vector Ad5/F35-mediated APE1 siRNA (Ad5/F35-siAPE1). The p53 mutant cell lines MHCC97L showed radioresistance, compared with HepG2 and Hep3B cells. APE1 was strongly expressed in MHCC97L cells and was induced by irradiation in a dose-dependent manner, and Ad5/F35-siAPE1 effectively inhibited irradiation-induced APE1 and p53 expression. Moreover, silencing of APE1 significantly potentiated the growth inhibition and apoptosis induction by irradiation in all tested human HCC cell lines. In addition, Ad5/F35-siAPE1 significantly enhanced inhibition of tumor growth and potentiated cell apoptosis by irradiation both in HepG2 and MHCC97L xenografts. In conclusion, down regulation of APE1 could enhance sensitivity of human HCC cells to radiotherapy *in vitro* and *in vivo*.

## Introduction

Hepatocellular carcinoma (HCC) is one of the most prevalent malignant diseases in the world [1]–[3]. Radiotherapy represents a major therapeutic option for HCC patients [4], but the efficacy of this therapy is limited by intrinsic radioresistance of the tumor cells. Ionizing radiation (IR) can result in lethal cell damage, which is correlated with DNA damage induction and repair [5]. The activity of the DNA damage repair pathway is the major factor leading to radioresistance in tumors, including hepatoma.

DNA-repair systems play an important role in protecting the genomic stabilization and integrity. However, an elevated DNA repair capacity in tumor cells is associated with drug or radiation resistance. The human apurinic/apyrimidinic endonuclease (hereafter, APE1) is a key enzyme in the DNA base excision repair (BER) pathway, which plays a critical role in repairing DNA damaged by irradiation [6], [7]. In addition to its DNA repair function, APE1 maintains a number of transcriptional factors including p53 by both redox-dependent and –independent mechanisms in their reduced and active state, thereby regulating their DNA-binding activity, influencing gene expression and maintaining genomic stability [8], [9].

In fact, the tumor suppressor p53 gene is activated in response to DNA damage and encodes a transcription regulatory protein that acts as a brake by inducing either cell cycle arrest or apoptosis, thereby preventing the propagation of genetically damaged cells and then maintaining genomic stability by its participation in stress-response pathways and DNA repair pathways [10]. If p53 is mutated, however, the cell with DNA damage can escape from apoptosis and turn into cancer cells [11]. To date, some studies have documented that p53 alterations are correlated with the sensitivity to radiotherapy in human HCC cells [12], [13]. As known that, the p53 gene is mutated in approximately 50% of hepatoma cells [14], and the mutant p53 (mutp53) proteins not only lose their tumor suppressive activities but often gain additional oncogenic functions that endow cells with growth and survival advantages, differences in radio-sensitivity [15], [16]. The transversion in codon 249 of p53 gene, which causes an arginine to serine (R→S) substitution is most commonly present in human HCC patients [17]. Mutated R249S p53 protein expression may induce cell proliferation and apoptosis inhibition [18], [19].

Several studies demonstrated that APE1 was overexpressed in several human tumors, such as osteosarcoma, colorectal cancer, ovarian cancer, cervical cancer, and non-small cell lung cancer [20]–[24]. In normal hepatocytes and endothelial and biliary duct cells, APE1 was detected only in nucleus of cells, and the shift of APE1 from nucleus to cytoplasm was observed in HCC cells. The expression of nuclear and cytoplasmic APE1 was significantly higher in HCC tissue than in the surrounding cirrhosis [25].Furthermore, more recent analysis showed that increased APE1 expression was associated with radioresistance. A decrease in APE1 levels led to enhanced cell sensitization to ionizing radiation in human osteogenic sarcoma cells and lung carcinoma cells as well as in colorectal cancer cells [22], [23], [26], [27].We have previously shown that APE1 was overexpression in human colorectal cancer, and chimeric adenoviral vector Ad5/F35-mediated APE1 siRNA (Ad5/F35-siAPE1) potentiates radiosensitivity of human colorectal cancer cells [23].

In this study, we explored the radiosensitivity profiles of human HCC cell lines by measuring cell survival and apoptosis in MHCC97L, HepG2 and Hep3B cells, and investigated the correlation existing between APE1 deficiency and the sensitivity of HCC cells to radiotherapy. Additionally, we tested whether the downregulation of APE1 protein could potentiate the inhibition of tumor growth by irradiation *in vivo*. The results provided by our study demonstrate that MHCC97L showed strongly resistance to irradiation, and Ad5/F35-siAPE1 could inhibit irradiation-induced APE1 and p53 expression. More importantly, the present study firstly demonstrated that Ad5/F35-siAPE1 enhanced sensitivity of human HCC cells to radiotherapy *in vitro* and *in vivo*.

## Materials and Methods

### Materials

DMEM and fetal bovine serum were from Invitrogen (Grand Island, NY, USA). Polyvinylidene difluoride (PVDF) transfer membrane was purchased from Sigma-Aldrich (St. Louis, MO, USA). The monoclonal antibody against hAPE1 was from Novus Biological (Littleton, CO, USA). All of the antibodies directed against p53 (DO-1), p21 and β-actin were purchased from Santa Cruz Biotechnology (Santa Cruz, CA, USA).

### Cell Lines

HepG2 (wtp53, carrying wild-type p53), Hep3B (p53 null, lacking p53) and MHCC97L (mutp53, harboring mutant p53) human hepatoma cell lines [28], [29] were obtained from the Cell Institute of Shanghai (Academia Sinica, Shanghai, China). Cells were maintained at 37°C in a humidified incubator under 5% CO_2_ and grown in Dulbecco’s modified Eagle medium (DMEM) supplemented with 10% fetal bovine serum, 50 mg/ml penicillin/streptomycin.

### Irradiation

For X-ray treatment, cells were cultured in six-well plates until they reached 75% confluence and then irradiated at 200 cGy/min, at room temperature, with an Elekta Precise Linear Accelerator operating at 8 MV.

### MTT Assay

Cells(1×10^5^ cells/ml) were immediately inoculated into 96-well plates (200 µl/well) in triplicate post-irradiation. After 72 h, 15 μ l MTT (5 g/l) was added to each well and incubated for 4 h, and then the culture medium was discarded followed by addition of 200 μ l DMSO and vibrated for 10 min. The OD value at 492 nm was determined using a microplate reader. Cell viability (%) = OD value of the treatment group/OD value of the control group×100%.

### Colony Formation Assay

Following irradiation, cells were counted, and plated in triplicate at a density to give between 30 and 300 colonies/10-cm dish. Cells were allowed to proliferate in culture media for 10∼14 days, with fresh media replacement every 3 days. Colonies were fixed and stained in 0.1% crystal violet in absolute ethanol for cell counting. Clones of at least 50 cells were counted as one colony. Survival curves were plotted as the log of survival fraction versus radiation dose.

### Assessment of Apoptosis by Annexin-V and PI Double-staining Flow Cytometry

Cells were treated with X-ray radiation in different doses as described above. At 48 h post-irradiation, the cells were harvested and then stained with annexin V-FITC and PI (Invitrogen). Then samples were analyzed by flow cytometry.

### Infections

Adenovirus vector Ad5/F35-siAPE1 carrying human APE1 siRNA sequence was constructed and purified as described previously [23]. The control adenovirus, Ad5/F35-EGFP, was purchased from Vector Gene Technology Company Limited (Beijing, China). HepG2, Hep3B and MHCC97L cell lines were infected with Ad5/F35-EGFP or Ad5/F35-siAPE1 for 2 hours and replaced with fresh medium. Cells were cultured for another 48 hours and then analyzed by Western blot and MTT assay or prepared for following experiments.

### Western Blot Analysis

Equal amounts of protein from nuclear or cytosolic extract or whole-cell lysate, were electrophoresed by 10% SDS–PAGE. Proteins were then transferred onto PVDF membranes. After being blocked in Tris-Buffered Saline and Tween 20 (TBST) (50 mM Tris-HCl, pH 7.5, 150 mM NaCl and 0.1% [volume/volume] Tween 20) containing 5% (weight/volume) defatted milk for 1 h at 37°C, membranes were incubated with the specific primary antibody. After three washes with TBST, the membranes were incubated for 1 h at 37°C with the appropriate peroxidase-conjugated secondary antibodies. Then, the membranes were washed three times with TBST and the blots were reacted with chemiluminescence reagents and revealed with Biomax-Light films (Kodak, Rochester, NY, USA). Band intensities were analyzed using the Gel Doc 2000 apparatus and software (Quantity One; Bio-Rad). Suppliers of incubation conditions for antibodies used for Western blot were as follows: anti-APE1 monoclonal (Novus), 1 h at 37°C, dilution 1∶5000; anti-p21 monoclonal antibody (Santa Cruz), overnight at 4°C, dilution 1∶500; anti-p53 monoclonal antibody (DO-1), overnight at 4°C, dilution 1∶500; anti-β-actin monoclonal (Santa Cruz), 1 h at 37°C, dilution 1∶2000.

### Quantitative RT-PCR

Total RNA was extracted by using Trizol (Invitrogen) and chloroform/isoamyl alcohol precipitation following the manufacturer’s instructions. RNA concentrations were determined by spectrophotometer (Eppendorf AG, Hamburg, Germany). Subsequently, 1 µg of total RNA were reverse transcribed into single-stranded DNA using SuperScript II (Invitrogen). Quantitative RT-PCR was performed using SYBR Premix Ex Taq (TaKaRa) in a LightCycler 480 real-time PCR system (Roche, Indianapolis, IN, USA). Primer sequences were: 5′-TTAGATTGGGTAAAGGAAGAAGC-3′ (forward), and 5′-CTGACCAGTATTGATGAGAGAGT-3′ (reverse) for APE1; 5′-GGAGGGGCGATAAATACC-3′ (forward) and 5′-AACTGTAACTCCTCAGGCAGGC-3′ (reverse) for p53; 5′-CTGGAGACTCTCAGGGTCGAAA-3′ (forward) and 5′-TTCTCCAAGAGGAAGCCCTAATC-3′ (reverse) for p21. Control PCR was performed using β-actin primer: 5′-GATCATTGCTCCTCCTGAGC-3′ (forward) and 5′-TGTGGACTTGGGAGAGGACT-3′ (reverse). Primer pairs for all detected genes were designed to yield 100- to 300-bp amplicons, which are suitable for real-time quantitation. Gene expression was determined by normalization against β-actin expression.

### In Vivo Experiments

All experiments were carried out in accordance with China Animal Welfare Legislation and were approved by the Third Military Medical University Committee on Ethics in the Care and Use of Laboratory Animals. HepG2 or MHCC97L cells (5×10^6^) in 100 µl phosphate-buffered saline (PBS) were injected subcutaneously into the right flank of nude mice, respectively. When the tumors grew to approximately 50 mm^3^ on day 7 after cell injection, 28 tumor-bearing mice were randomized into the following four treatment groups (n = 7 animals per group): (a) Ad5/F35-EGFP; (b) Ad5/F35-siAPE1; (c) Ad5/F35-EGFP+IR; (d) Ad5/F35-siAPE1+IR. Mice were injected directly into the tumors with Ad5/F35-EGFP or Ad5/F35-siAPE1. Two days later, tumors in groups (c) and (d) were irradiated with 6 Gy of X-ray. On day 16, xenografts from each group were completed isolated and tumor volumes were then examined exactly.

The maximum diameters (*Dmax*) and minimum diameters (*Dmin*) of xenografts were measured before each treatment and after mice killed, and tumor size was calculated according to the formula: tumor size (mm^3^) = (*Dmax*×*Dmin* ^2^)/2. From the tumor growth curves, tumor-doubling time (DT) was determined for each individual tumor. Tumor growth delay was calculated by subtracting the mean tumor volume doubling time of the untreated tumors (control) from the mean tumor volume doubling time of each experimental group. Specific growth delay (SGD) was calculated according to the formula: SGD = (T_2_−T_1_)/T_1_; where T_1_ is the time taken in days for control tumors and T_2_ is the time for treated tumors to double in volume. Inhibition ratio, expressed in percent, was calculated at day 16 after mice killed by the formula [1-(treated tumor average volume/untreated tumor average volume)]×100%.

### Immunohistochemical Analysis of Tumors for Ki67

Sections from paraffin-embedded tumors were incubated with Ki67 antibody (clone MIB-1; Dako) overnight at 4°C. Sections were rinsed with PBS and incubated with goat anti-mouse secondary antibody. Sections were rinsed with PBS and developed with diaminobenzidine substrate, and then counterstained with diluted Harris haematoxylin. Ki67 staining was quantified using computer-assisted image analysis with Image Pro Plus software (Media Cybernetics). The image analysis was done on four random fields (magnification,×100) per section from a total of five sections per group.

### In situ Apoptosis Detection by TUNEL Staining

The formalin-fixed and paraffin-embedded 5 µm-thick sections of all tumor samples were analyzed for apoptosis by terminal dUTP nick end labeling (TUNEL) staining using the Apoptag Kit (Intergen, Purchase, NY, USA). The extent of apoptosis was evaluated by counting the positive brown-stained cells as well as the total number of cells at 10 arbitrarily selected × 100 microscope fields in a blinded manner.

### Statistical Analysis

All quantitative data were obtained from three independent experiments and expressed as mean ± standard deviation values. The statistical significance of differences was determined by one-way analysis of the variance (ANOVA) using computer SPSS software SPSS 10.0 (SPSS, Chicago, IL, USA). A value of P<0.05 was considered statistically significant.

## Results

### Radiosensitivity of Human HCC Cell Lines

To examine the sensitivity of human HCC cell lines to radiotherapy, MTT and colony formation assays were performed on HepG2, Hep3B and MHCC97L cells treated with various doses (0∼10 Gy) of radiation at 48 h post-irradiation. MTT assay showed that a significantly increased cell survival was observed in MHCC97L cells, compared with HepG2 or Hep3B cells (Fig. 1A). In addition, Fig. 1A showed that the cell survival in Hep3B cells after irradiation at 4, 6, 8 or 10 Gy dose was higher than that in HepG2 cells. Because MTT assay was an overall measure of cell viability and was not necessarily indicative of long-term cell survival and proliferation, a clonogenic survival assay also was used. Fig. 1B reveals that cell colonies at all tested doses of radiation significantly increased in MHCC97L cells, compared with HepG2 or Hep3B cells. Moreover, the cell colonies in Hep3B cells after irradiation at 4, 6, 8 or 10 Gy dose significantly increased, compared with HepG2 cells (Fig. 1B).

**Figure 1:** Dose-dependent growth inhibition of three human HCC cells with different p53 status. Cell survival following exposure to various doses of X-ray was evaluated by MTT assay (A) and colony formation assay (B). The values are expressed as the mean±standard deviation from three independent experiments.

To investigate the apoptosis induction effect by radiation *in vitro* in human HCC cells, cells were treated with different doses (0, 4 or 10 Gy) of radiation, stained with annexin V-FITC and PI, and analyzed by flow cytometry at 48 h post-irradiation. Significantly decreased apoptotic cells at 10 Gy of radiation were observed in MHCC97L cells, compared with HepG2 and Hep3B cells, but there are no significant differences of apoptotic cells between MHCC97L and Hep3B cells at 4 Gy (Fig. 2). In addition, the apoptotic cells in Hep3B after 4 or 10 Gy irradiation were lower than that in HepG2 cells (Fig. 2). Therefore, these results meant that the sensitivity of MHCC97L cells to radiotherapy was lower than that of HepG2 and Hep3B cells, and Hep3B cells were much more radioresistant compared to HepG2 cells.

**Figure 2:** Dose-dependent apoptosis induction in three human HCC cell lines irradiated with X-rays. Each data point represents the mean±standard deviation of three independent determinations. ^*^P<0.05, ^**^P<0.01 vs HepG2 cells; ^#^P<0.05 vs Hep3B cells.

### APE1 is Induced by Irradiation in a Dose-dependent Manner in MHCC97L Cells

We have determined that MHCC97L cells were less sensitive to irradiation compared to HepG2 and Hep3B cells. To investigate the role of APE1 in sensitivity of MHCC97L cells to radiotherapy, we analyzed the protein expression of APE1 at 48 h post-irradiation by western blotting. A dose-dependent increase in APE1 protein expression in MHCC97L cells was observed post irradiation (Fig. 3A and B), possibly promoting radioresistance. The APE1 protein expression in 6 Gy irradiation group was much higher than that in high dose (8 or 10 Gy) X-ray irradiation group, which may due to the high-dose induced cell death in MHCC97L cells.

**Figure 3:** APE1 is induced by X-ray radiation in a dose-dependent manner in MHCC97L cells. Western blot analysis of cell lysates for the protein expression of APE1 at 48 h post irradiation. Normalized APE1 protein levels after adjusting for loading. *P<0.05, **P<0.01 vs control.

### Ad5/F35-siAPE1 Suppresses APE1-target Gene Expression and Inhibits Irradiation-induced APE1 Expression

To determine the combined effect of APE1 silence and irradiation, western blotting and qRT-PCR were performed on MHCC97L cells. A significant decrease in APE1 and P53 protein expressions was observed at 48 h after Ad5/F35-siAPE1 infection in MHCC97L cells, whereas there was no P21 protein expression in all tested groups (Fig. 4A). Interestingly, we also found that irradiation-induced APE1 and P53 expressions were almost completely inhibited by the pretreatment of cells with Ad5/F35-siAPE1 (Fig. 4A). The mRNA expressions of APE1, P53 and P21 decreased in Ad5/F35-siAPE1 group, and irradiation-induced expressions of APE1 and APE1-target genes mRNA were significantly suppressed by Ad5/F35-siAPE1 pretreatment (Fig. 4B).

**Figure 4:** Ad5/F35-siAPE1 inhibits irradiation-induced APE1 expression. (A) MHCC97L cells were treated with Ad5/F35-siAPE1 or Ad5/F35-EGFP; cells were irradiated with 6 Gy of X-ray at 48 h post-infection, and the APE1, p53 and p21 protein expressions were determined at 48 h post irradiation by western blot. Normalized APE1, P53 and P21 protein levels after adjusting for loading. (B) Quantitative RT-PCR reaction target gene analysis was similarly performed in MHCC97L cells. Each data point represents the mean ± standard deviation of three independent determinations.^ *^P<0.01 vs Ad5/F35-EGFP; ^#^P<0.01 vs Ad5/F35-EGFP+IR.

### Ad5/F35-siAPE1 Enhances Cell Growth Inhibition and Apoptosis Induction by Irradiation In Vitro

We investigated the effect of Ad5/F35-siAPE1 combined with radiotherapy on human hepatoma cell lines, MTT and colony formation assays were employed. HepG2, Hep3B and MHCC97L cells were treated with an empty adenoviral vector (Ad5/F35-EGFP) or Ad5/F35-siAPE1, and then irradiated with various doses (0∼10 Gy) of radiation. Significantly decreased cell survival was observed in Ad5/F35-siAPE1+IR group compared to Ad5/F35-EGFP+IR group at all tested doses of radiation in HCC cells, respectively (Fig. 5A). As shown in Fig. 5B, significantly decreased cell colonies at all tested doses of irradiation in HCC cells were observed in Ad5/F35-siAPE1 group when compared with Ad5/F35-EGFP group, which indicates a protective effect of APE1 on IR-induced apoptosis. Although there were no significant differences in Ad5/F35-siAPE1+IR induced cell growth inhibition in HCC cell lines, the results suggest that Ad5/F35-siAPE1 enhanced sensitivity of mutp53 cells to radiotherapy as well as wtp53 and p53 null cells.

**Figure 5:** Ad5/F35-siAPE1 enhances cell killing following irradiation in human HCC cell lines. Cells were infected with Ad5/F35-EGFP or Ad5/F35-siAPE1. At 48 h post-infection, samples were treated with different doses of irradiation. Cell survival following exposure to various doses of irradiation was evaluated by MTT (A) and colony formation assay (B). Each data point represents the mean±standard deviation of three independent determinations. Significant differences existed at all doses levels at the P<0.05 level.

To examine the effects of Ad5/F35-siAPE1 on apoptosis induction by irradiation *in vitro*, cells were stained with annexin V-FITC antibody and PI, and analyzed by flow cytometry. As shown in Fig. 6, the number of apoptotic cells in Ad5/F35- siAPE1-transfected group was much more than that of Ad5/F35-EGFP-transfected group at 4 and 10 Gy doses radiation in all tested HCC cell lines (HepG2∶17.45 vs 12.16, 28.11 vs 20.08; Hep3B: 15.22 vs 10.65, 23.35 vs 16.32; MHCC97L: 13.75 vs 9.09, 20.54 vs 12.59). Compared to Ad5/F35-EGFP control group, the percentage of apoptotic cells in Ad5/F35-siAPE1 group increased by 63.15% at 10 Gy of radiation in MHCC97L cells, which was much higher than that in HepG2 (39.99%) and Hep3B (43.08%) cells. Thus, these results demonstrate that silencing of APE1 by Ad5/F35-siAPE1 enhanced the apoptosis induction by irradiation in HCC cells.

**Figure 6:** Cell apoptosis following combined treatment with Ad5/F35-siAPE1 and irradiation *in vitro*. HepG2, Hep3B and MHCC97L cells were treated with Ad5/F35-EGFP or Ad5/F35-siAPE1.Samples were collected at 48 h for a range of X-ray irradiation (0, 4 and 10 Gy). At another 48 h post-irradiation, the cells were harvested and then stained with annexin V-FITC and PI. Bar graphs represent the mean values of triplicate determinations ± standard deviation. *P<0.01 vs Ad5/F35-EGFP.

### Ad5/F35-siAPE1 Potentiates the Inhibition of Tumor Growth by Irradiation In Vivo

We have shown that Ad5/F35-siAPE1 enhances cell growth inhibition by irradiation in human hepatoma cells *in vitro*. To investigate whether Ad5/F35-siAPE1 could potentiate the inhibition of tumor growth by irradiation *in vivo*, tumor-bearing mice were injected intratumorally with Ad5/F35-EGFP or Ad5/F35-siAPE1, and two days later tumors were irradiated with 6 Gy of X-ray. Fig. 7A shows that Ad5/F35-siAPE1 combined with irradiation caused a significant inhibition of tumor growth compared with Ad5/F35-EGFP+IR or Ad5/F35-siAPE1 alone in HepG2 xenografts. On day 16, the tumor-inhibition rates of Ad5/F35-siAPE1 group, Ad5/F35-EGFP+IR group and Ad5/F35-siAPE1+IR group were 30.5, 28 and 74.65% (Fig. 7A and Table 1), respectively (P<0.05). As shown in Fig. 7B and Table 1, the results showed that the tumor-inhibition rates of Ad5/F35-siAPE1 group, Ad5/F35-EGFP+IR group and Ad5/F35-siAPE1+IR group at day 16 were 29.56, 25.76 and 72.15% in MHCC97L xenografts, respectively (P<0.05). As shown in Table 1, treatment with Ad5/F35-siAPE1 or irradiation alone significantly delayed HepG2 xenografts regrowth, however, only Ad5/F35-siAPE1 alone significantly delayed MHCC97L xenografts regrowth, whereas treatment with irradiation alone did not delay MHCC97L xenografts regrowth. More importantly, the combination of Ad5/F35-siAPE1 and irradiation significantly increased the delay of HepG2 and MHCC97L xenografts regrowth compared with that produced by Ad5/F35-siAPE1 or irradiation alone (Table 1).

**Figure 7:** *In vivo* evaluation of tumor growth in human hepatoma wtp53 and mutp53 xenografts. Tumor-bearing mice were injected directly into the tumors with Ad5/F35-siAPE1 or Ad5/F35-EGFP at the 1,6,11th day. Two days later, tumors were irradiated with 6 Gy of X-ray. Tumors were assessed for growth by measuring the volume of xenografts. (A) Tumor volume of HepG2 xenograft. (B) Tumor volume of MHCC97L xenograft.

**Table 1:** Tumor growth after treatment with single factor (Ad5/F35-siAPE1 or irradiation) or combination on hepatoma tumor model.

	HepG2 xenografts					MHCC97L xenografts			
Experimental groups		N	DT (days) Mean±SD	SGD Mean±SD	Inhibitionratio (%)	N	DT (days) Mean±SD	SGD Mean±SD	Inhibitionratio (%)
Ad5/F35-EGFP		4	3.48±0.13			4	3.56±0.17		
Ad5/F35-siAPE1		4	3.9±0.1	0.12±0.07	30.5	4	4.09±0.06	0.15±0.07	29.56
Ad5/F35-EGFP+IR		4	3.86±0.14	0.11±0.07	28	4	3.9±0.11	0.1±0.07	25.76
Ad5/F35-siAPE1+IR		4	6.1±0.47	0.75±0.08	74.65	4	5.73±0.16	0.61±0.07	72.15

IR = irradiation; N = number of mice in the experimental group; DT = tumor doubling time; SGD = specific growth delay.

To further investigate cell growth inhibition of Ad5/F35-siAPE1 by irradiation, Ki67 immunohistochemistry was performed on human hepatoma xenografts. As shown in Fig. 8A, the Ki67^+^ nuclei in Ad5/F35-siAPE1+IR group were lower than that in Ad5/F35-siAPE1 or Ad5/F35-EGFP+IR group alone. As in MHCC97L xenografts, Fig. 8B also shows that Ad5/F35-siAPE1 in combination with irradiation caused a significant inhibition of proliferating cell numbers compared with Ad5/F35-siAPE1 or Ad5/F35-EGFP+IR alone. However, no significant difference was observed between Ad5/F35-siAPE1 and Ad5/F35-EGFP+IR groups. The results further reveal that Ad5/F35-siAPE1 enhanced the cell growth inhibition by irradiation in human hepatoma xenografts.

**Figure 8:** Combined treatment with Ad5/F35-siAPE1 and irradiation in tumor cell proliferation *in vivo*. HepG2 or MHCC97L cells were treated with Ad5/F35-siAPE1 or Ad5/F35-EGFP; 48 h after infection, cells were irradiated (6 Gy), and tumor cell proliferation was assessed by Ki67 immunohistochemistry. (A) Immunohistochemistry of HepG2 xenograft. (B) Immunohistochemistry of MHCC97L xenograft. Each data point represents the mean±standard deviation of three independent determinations. Lane 1, Ad5/F35-EGFP; lane 2, Ad5/F35-siAPE1; lane 3,Ad5/F35-EGFP+IR; lane 4, Ad5/F35-siAPE1+ IR. ^*^P<0.01 vs Ad5/F35-EGFP; ^#^P<0.01 vs Ad5/F35-siAPE1; ^$^P<0.01 vs Ad5/F35-EGFP+IR.

### Ad5/F35-siAPE1 Enhances the Apoptosis Induction by Irradiation In Vivo

To investigate the effect of Ad5/F35-siAPE1 on apoptosis induction by irradiation in HepG2 and MHCC97L xenografts, we measured apoptotic cells by TUNEL assay. We found that a much higher apoptosis index was observed in the Ad5/F35-siAPE1+IR group compared with Ad5/F35-EGFP control group, Ad5/F35-EGFP+IR group or Ad5/F35-siAPE1 group in HepG2 xenografts (Fig. 9A). Then, we investigated whether silencing of APE1 could potentiate the apoptosis induction by irradiation in MHCC97L xenografts, and found that Ad5/F35-siAPE1 increased significantly cell apoptosis induction by irradiation (Fig. 9B).

**Figure 9:** Combined treatment with Ad5/F35-siAPE1 and irradiation induces apoptosis *in vivo*. HepG2 or MHCC97L cells were treated with Ad5/F35-siAPE1 or Ad5/F35-EGFP; 48 h after infection, cells were irradiated (6 Gy), and apoptosis was determined at 24 h post irradiation by terminal dUTP nick end labeling (TUNEL) staining. (A) TUNEL staining of HepG2 xenograft. (B) TUNEL staining of MHCC97L xenograft. Data are expressed as percentage of apoptosis-positive cells examined with TUNEL. Bar graphs represent the mean values of triplicate determinations ± standard deviation. Lane 1, Ad5/F35-EGFP; lane 2, Ad5/F35-siAPE1; lane 3,Ad5/F35-EGFP+IR; lane 4, Ad5/F35-siAPE1+ IR.^ *^P<0.01 vs Ad5/F35-EGFP; ^#^P<0.01 vs Ad5/F35-siAPE1; ^$^P<0.01 vs Ad5/F35-EGFP+IR.

## Discussion

Human hepatocellular carcinoma (HCC),one of the most common lethal malignant diseases worldwide, is responsible for a large number of deaths annually [30]. Surgery and radiotherapy are two commonly used treatment modalities for HCC. Although surgical resection offers a good therapeutic effect and low risk of complication, only 15% of the patients are eligible for optimal resection at diagnosis. Radiotherapy represents a major therapeutic option for HCC patients, but its efficacy is limited by the inherent tumor radioresistance and low radiation tolerance of the surrounding normal liver [31]. Therefore, researches that overcome tumor resistance to radiotherapy and reduce normal tissue complications are urgently needed. To improve the therapeutic efficacy, there has been much interest in using of radiosensitizers in combination with radiotherapy [22], [23], [32].

DNA-repair systems are important in maintaining genomic stabilization and integrity. However, an elevated DNA repair capacity in cancer cells leads to drug or radiation resistance. Therefore, reducing the DNA repair capability of cancer cells could enhance the efficacy of these agents. DNA repair proteins are becoming fundamental targets for enhancing cancer therapy [33]–[35]. In particular, APE1 is becoming a leading target due to its central involvement in DNA base excision repair (BER) pathway, which accounts for nearly all of the abasic site cleavage activity in most cultured human cell lines [36]. APE1 is also thought to interact with several proteins including 8-oxoguanine DNA glycosylase, X-ray cross-complementing-1, DNA polymerase β, proliferating cell nuclear antigen and flap endonuclease 1 [37]. Moreover, APE1 has 3′-repair diesterase or phosphatase activity, which is important in repairing DNA that has been damaged by radiation. In addition to its DNA repair functions, APE1 exerts its reduction–oxidation (redox) modification activity on some transcriptional factors, and regulates their DNA-binding activity, and thereby, regulate gene expression [38]. p53 is an important tumor suppressor that helps maintain genomic stability by its participation in many DNA repair pathway [39], [40]. The previous studies showed that APE1 was responsible for reducing p53, thus enhancing its DNA-binding activity [8], [9]. Since APE1’s redox constitutively influences on p53, APE1 contributes to p53’s DNA repair activities.

The present study found that the radiosensitivity of MHCC97L mutp53 cells was lower than that of Hep3B p53 null and HepG2 wtp53 cells, which is in accord with the previous studies [12], [13]. Given that the mutp53 proteins not only lose wtp53 tumor suppressor activities, but also gain new oncogenic properties favoring cancer development [41], our observations suggest a key role of mutp53 involved in the cellular response to irradiation. Furthermore, our investigations provide a dose-dependent growth inhibition and apoptosis induction by irradiation for hepatoma cell lines and mutp53 cells provide much more resistance to radiotherapy than p53 null and wtp53 cells, which giving far more detailed information. Moreover, our results also showed that the radiosensitivity of HepG2 cells was higher than that of Hep3B cells. Taken together, the loss or mutation of p53 proteins produced radioresistance, which is in line with other studies showing that p53 is essential in regulating the radiosensitivity of mammalian cells [13], [42].

APE1 expression has been found to be associated with radioresistance in tumors [22], [23], [26], [27]. However, very few data exist on APE1 expression and response to irradiation in HCC. The present study found that APE1 was strongly expressed in MHCC97L cells and irradiation resulted in APE1 accumulation, probably representing an early event in the cell response to irradiation because of its role in DNA BER. Furthermore, Ad5/F35-siAPE1 inhibited APE1 expression and AP endonuclease activity (Figure S1), which suggests that Ad5/F35-siAPE1 would potentiate irradiation-induced DNA damage and suppress DNA repair. Loss or inhibition of p53 provided resistance to radiotherapy, which shows that p53 has been linked to radioresistance in tumor cells [13], [42]. p53 not only promotes the repair of minor DNA damage induced by radiation but also induces apoptosis of cells with severe DNA damage [43]. Failure of this p53-dependent apoptosis procedure may result in genomic instability after irradiation [44]. In this study, the radioresistance of mutp53 cells was higher than that of wtp53 cells, which is in line with the previous research [13], indicating that mutp53 gain new properties related to radiotherapy.

Several studies demonstrated a high expression in several human tumors, such as cervical cancer [20], ovarian cancer [21] and osteosarcoma [22]. Furthermore, more recent study shows that APE1 expression levels are correlated with sensitivity of cancer cells to radiotherapy and chemotherapy, and APE1 inhibitor could enhance the efficacy of conventional cancer treatment such as radiotherapy. Our previous study has demonstrated that vector-based APE1 siRNA decreased APE1 protein expression, and enhanced the chemosensitivity of multiple myeloma to melphalan [45] and radiosensitivity of human colorectal cancer [23]. In this study, combined treatment with Ad5/F35-siAPE1 and irradiation not only enhanced the cell growth inhibition and apoptosis induction, but also increased the tumor-doubling time, specific growth delay and tumor-inhibition ratio (%). The present study is the first to confirm that silencing of APE1 by adenoviral vector Ad5/F35-mediated APE1 siRNA enhanced sensitivity of human HCC cells to radiotherapy *in vitro* and *in vivo.* Therefore, inhibition of APE1 protein by APE1-specific siRNA may be a strategy to overcome radioresistance and then improve its therapeutic efficacy for hepatoma. Furthermore, the clinical use of Ad5/F35-APE1 siRNA in combination with radiotherapy is unexplored to date and yet important to investigate in human HCC patients.

## Supporting Information

Figure S1 **Effects of combined Ad5/F35-siAPE1 and irradiation on AP endonuclease activity.** HepG2 and MHCC97L cells were treated with Ad5/F35-EGFP or Ad5/F35-siAPE1; 48 h after infection, cells were irradiated (6 Gy) and AP endonuclease activity of cell lysates was examined at 48 h post irradiation by oligonucleotide cleavage assay. The data indicated that the AP endonuclease activity of cell lysates was drastically decreased in Ad5/F35-siAPE1 group. Meanwhile, Ad5/F35-siAPE1 inhibited irradiation-induced AP endonuclease activity.
(TIF)

Text S1 **Supporting information materials and methods.**
(DOCX)
